The article "The Effect and Related Mechanism of Action of Astragalus Compatible with Curcumin against Colon Cancer Metastasis in Mice" was retracted in 2023. Reasons: signs of a paper mill; suspected computer-generated content; unreliable results or conclusions; concerns about the data.

# The Effect and Related Mechanism of Action of Astragalus Compatible with Curcumin against Colon Cancer Metastasis in Mice

**DOI:** 10.1155/2022/9578307

**Published:** 2022-06-10

**Authors:** Jiafei Wu, Decai Tang

**Affiliations:** School of Traditional Chinese Medicine and School of Integrated Chinese and Western Medicine, Nanjing University of Chinese Medicine, Nanjing, 210046 Jiangsu, China

## Abstract

Colon cancer (CC) is the third most common tumor worldwide. Colon carcinogenesis is strongly linked to inflammation. The initiation and progression of colon cancer may be influenced by epigenetic processes. Cancer metastasis is a multistep process involving several genes and their products. During tumor metastasis, cancer cells first enhance their proliferative capacity by lowering autophagy and apoptosis, and then, their capacity is stimulated by boosting tumors' ability to take nutrients from the outside via angiogenesis. Traditional treatment focuses on eliminating tumor cells by triggering cell death or activating the immune system, which often results in side effects or chemoresistance recurrence. On the contrary, Chinese medicine theory considers the patient's entire inner system and aids in tumor shrinkage while also taking into account the mouse' general health. Because many Chinese herbal medicines (CHM) are consumed as food, using edible CHMs as a diet resource therapy for colon cancer treatment is a viable option. Two traditional Chinese herbs, Astragalus membranaceus and Curcuma zedoaria, are commonly utilized jointly in colon cancer preventive therapy. As a result, the anticancer effect of astragalus and curcumin (AC) on colon cancer suppression in an 18-week AOM-DSS colon cancer mouse model is investigated in this research. These findings may offer a scientific foundation for investigating colon cancer diagnostic biomarkers and therapeutic application of AC in colon cancer treatment. These studies also highlighted the potential effect and mechanism of AC in the treatment of colon cancer, as well as providing insight into how to effectively use it.

## 1. Introduction

Colon cancer is a common malignant tumor illness, which progresses to be a leading reason of cancer-associated mortalities across the world. Colon cancer is caused by inadequate exercise, moderate alcohol use, old age, family background, high-fat diets with minimal nutrition and red meat, diabetes, and inflammatory conditions such as peptic ulcer and Crohn's disease. Whereas most malignancies are rare, some are hereditary, like those caused by mutations in the APC gene in chronic granulomatous primary sclerosing coli or mutations in the MMR machinery genes in Lynch syndrome. Colitis-related tumor is a lifelong complication of irritable bowel syndrome that can occur in both Crohn's disease and psoriatic arthritis with colonic inclusion. Furthermore, ecological variables and lifestyle-associated elements like obesity, inactivity, and smoking have been linked to an increased risk of colon cancer [1]. The dried roots of Astragalus membranaceus (AM) is utilized to cure common colds, diarrhea, weariness, and anorexia. Saponins, flavonoids, and polysaccharides are some of the energetic components of AM. AM's antioxidation, anti-inflammation, and immune system reaction boosting effects have been proven in pharmacological trials. AM shall be a possible anticancerous agent, according to mounting data. AM, for example, has been shown to prevent rat hepatocarcinogenesis. Tumor growth suppression, tissue invasiveness and angiogenesis reduction, and apoptosis induction have all been examined extensively using Astragalus saponins. 5-FU coupled with Astragalus polysaccharides improves the chemosensitivity of hepatoma tissues in combination therapy [2].

The development and/or metastasis of certain forms of cancer have been inhibited by specific Chinese herbs or formulations. Many of the herbs' active constituents may directly suppress cancer growth when isolated from the plants themselves as a whole. However, the most often utilized approach in the clinic is a Chinese herbal compound formula, which is more successful when various herbs and specific proportions are utilized jointly in specific combinations. The link between compatibility and impact shall, therefore, be studied in order to learn more about the compatibility or proportion of already known and undiscovered energetic components. HQ and EZ are two herbs often utilized in TCM for the treatment of various malignancies [3]. Natural compounds separated from the Curcuma genus are broadly employed in cooking around the world, as well as being traditionally prescribed for a wide range of ailments, including inflammation and fever, as well as for the avoidance and therapy of cardiovascular and malignant infections, primarily in Asian nations. However, there are many different species of the plant in the Curcuma genus, and several compounds have been extracted, including the active ingredient curcumin (as well as other curcuminoids and turmeric). Their antioxidant, anti-inflammatory, and antitumor properties have all been studied extensively [4]. New antitumor therapeutic compounds discovered in Chinese materia medica (CMM) have lately garnered attention since they are useful for boosting effectiveness, controlling the body's immunological operation, and minimizing drug resistivity. As a result, they are less likely to cause hazardous side effects. Clinical investigations have shown that the traditional medication mixture of Astragalus membranaceus-Curcuma (AC), initially described in “Yixuezhongzhongcanxilu,” is effective against gastrointestinal inflammation as well as several cancers. A rigorous investigation of AC's anticolorectal effects and the ideal dose ratio has yet to be conducted, and the underlying mechanisms remain obscure [5].

The impact and related mechanism action of astragalus compatible with curcumin against colon cancer metastasis in mice is analyzed in this work. The remainder of this paper is arranged as follows. The literature pieces related with this study are presented in Section 2. The suggested model is explained in Section 3. The findings and explanation of the proposed works are presented in Section 4. Eventually, Section 5 brings the paper's underlying theme to a conclusion.

## 2. Related Works

Reference [6] examined the significance of Azoxymethane/Dextran sodium sulphate as part of a well-established model of colitis-associated malignancy. When we looked at the animals after 12 weeks, we found that regardless of their genotype, they all had intestinal tumors. There were considerably more intestinal neoplasms in Dcn/mice than in wild-type mice in the microenvironment. Specifically, we discovered that the intestinal epithelium of Dcn/animals increased significantly in protein levels of factors linked with the epithelial-mesenchymal transition, such as Snail, Slug, Twist, and MMP2, under baseline settings that were not challenged. Dcn-deficient animals developed colitis-related cancer and in tandem with markers linked with the epithelial-mesenchymal transition (EMT). A combination of Celecoxib and decorin therapy showed encouraging results in treating human colorectal tumor tissues in decorin-deficient mice. A protein-based therapy, such as recombinant decorin treatment, has been developed to target the tumor microenvironment as a consequence of our findings, which give insight into colorectal cancer growth. There is now an increase in the use of patient-derived organoids as predictors of therapy responses, as well as molecular stratification of cancers, which forecast outcomes and therapy responses, and animal frameworks of metastatic illness [7]. A preclinical investigation was conducted to verify the Chinese Pharmacopoeia suggested doses of SB water extract for the treatment of colon cancers. [8]. Scutellaria barbata (SB) is a plant often used in cancer herbal remedies. UPLC was used to measure the scutellarin content in SBW. SBW or scutellarin was administered orally to mice with human HCT116 xenografts or murine colon tumors for four weeks. Human xenograft weights were lowered by 28.7, 36.9, and 28.8 percent, correspondingly, by SBW and scutellarin therapies. SBW and scutellarin treatments reduced lung metastases by 23.4 and 29.5 percent, correspondingly. This study showed evidence that SBW might have anticancer and antimetastatic impacts in colon tumor animal frameworks when administered at the mouse equivalent levels to the human dosages advised by CP. HOXC6's putative carcinogenic function and precise molecular mechanism in RCC were investigated in [9]. Overexpression of HOXC6 in RCC was shown to be related with a poor prognosis in this investigation. Colon cancer cells' motility and invasion were enhanced by HOXC6 overexpression, which activated the Wnt/-catenin signaling pathway and inhibited the release of DKK1. The translational impact of HOXC6 was also investigated and discovered that silencing HOXC6 increased the sensitivity of HCT116 and HT29 cells to irinotecan. Ileal immune profiles have been linked to colon cancer prognosis and treatment response [10]. Colonic immunity in both healthy and cancerous regions was downregulated in poor-prognosis cancer patients, except for the Th17 fingerprint of the ileal transcriptome, which was elevated in these individuals. There was a correlation between carcinogenesis and ileal inflammation in experimental frameworks of implanted and spontaneous mouse colon tumor, which was shown to be true across all of the studies. In contrast, oxaliplatin-dependent chemotherapies may restore a favourable, attenuated ileal immunological fingerprint in patients who respond to treatment. These findings imply that chemotherapy alters the ileum–tumor axis' immunological composition in a way that affects patient outcomes. “PD-relevant TIME” and the course of Parkinson's disease may be affected by MDSCs, according to one theory [11]. In order to test this theory, we used PD mice as a model system. Because the immune cells in the PD nodules were so few, we chose to look at the peritoneal cavity rather than the PD nodule when assessing the PD-relevant TIME. This resulted in a significant increase in intraperitoneal PMN-MDSCs as a consequence of PD progression. On the basis of these findings, we were able to demonstrate the utility of CD244 in identifying PMN-MDSCs phenotypically and functionally. Both interleukin-6 and granulocyte-colony stimulating factor levels in the peritoneal cavities were considerably elevated that is likely to have contributed to the rise in PMN-MDSCs. [12] In vitro and in vivo investigations show that LDEs have a significant role in the aetiology of IBD and CRC and that their therapy enhances the severity of colitis. To control the onset of IBD and CRC, we will look at how LDEs influence IBD and CRC development, as well as lifestyle variables that may have an impact on tissue levels of LDEs. Studying if the antitumor impact of a medication pair is different in various ratios, a colon cancer orthotopic transplantation model in mice was developed. For the purpose of determining the ideal ratio of Astragali Radix-Curcumae Rhizoma for the anticolon cancer action, PCA and CA were employed to investigate the tumor development and metastasis of the medication pair. Body weight, tumor volume, and number of liver metastases in colon cancer mice were measured after 15 days of treatment; pathological alterations in tumor tissue and liver tissue were noted by HE staining, as well. To monitor protein expression levels of tumor growth-related indicators in tumor tissue (Ki67, HBP1, and AFP), as well as tumor metastasis-related indicators in the liver tissue (E-cadherin, vimentin, and p53), the Western blot technique was utilized [13]. Astragali Radix-Curcumae Rhizoma's optimum anticolon cancer ratio was determined using PCA and CA. Various Astragali Radix-Curcumae Rhizoma ratios reduced tumor development and metastasis to variable degrees, according to the findings of the research. Tumor development was inhibited best by the Astragali Radix-Curcumae Rhizoma ratio of 1 : 1, while liver metastasis was inhibited best by the 2 : 1 ratio group, which improved weight loss. While the protein expression of HBP1 in tumor tissue of colon cancer mice was significantly upregulated by Astragali Radix-Curcumae Rhizoma, Ki67 and AFP in tumor tissue were significantly downregulated. When comparing the Astragali Radix-Curcumae Rhizoma compatibility groups, PCA showed that the closest groups to the sham operation group were in the range of 2 : 1, 1 : 1, and 3 : 2, with the closest group in the range of 2 : 1 having a distance from the control group of 2 : 1, which is in line with the commonly used clinimetric ratio of 2 : 1. Consistent with our theories, our CA findings indicated 11 different groups of colon cancer mice could be categorized as either being compatible with Astragali Radix-Curcumae Rhizoma or being sham operations. Clinical trials based on the findings of this research might lead to more successful use of Astragali Radix-Curcumae Rhizoma in the treatment of colon cancer. Combining p53 loss with AOM enhances tumor growth, including invasive malignancy and lymph node metastases. Reference [1] investigated this relationship. Colorectal tumor development and metastasis are also examined, including cell separation and coculture investigations, higher-resolution endoscopes, light-sheet fluorescence microscopy, and micro-CT imaging in mouse, as well as examination of partial epithelial-mesenchymal transition. For our protocol, we are looking for scientists who want to investigate factors that influence tumor formation in spontaneous or inflammation-driven conditions, including local invasiveness and lymph node metastasis. Preclinical in vivo analysis of new medications and other interventional methods for medical translation, as well as the assessment of developing imaging appliances, may be done in this environment. It may be finished in 10 weeks or 24 weeks if you follow Step 5A/C (using Step 5B). In colon tumor growth and metastasis, a decorin-deficient tumor microenvironment was shown to be important [14]. Adult wild-type and Dcn/- mice were given Azoxymethane/Dextran sodium sulphate as part of a well-established model of colitis-associated malignancy. When we looked at the animals after 12 weeks, we found that regardless of their genotype, they all had intestinal tumors. There were considerably more intestinal neoplasms in Dcn/mice than in wild-type mice in the microenvironment. Specifically, we discovered that the intestinal epithelium of Dcn/animals increased significantly in protein levels of factors linked with the epithelial-mesenchymal transition, such as Snail, Slug, Twist, and MMP2, under baseline settings that were not challenged. Dcn-deficient animals developed colitis-related cancer, and we observed that intercellular adhesion molecule 1 also enhanced, in tandem with markers linked with the epithelial-mesenchymal transition (EMT). A combination of Celecoxib and decorin therapy showed encouraging results in treating human colorectal tumor tissues in decorin-deficient mice. A protein-based therapy, such as recombinant decorin treatment, has been developed to target the tumor microenvironment as a consequence of our findings, which give insight into colorectal cancer growth. In vivo detection of micrometastases with specific chemotherapeutic efficacy by an intraoperative theranostic method use a tiny multifunctional drug [15]. CBHAc enabled very sensitive and selective real-time fluorescence diagnostic for zebra fish microtumors and mouse hepatic micrometastases by combining HDACs targeting with pH-responsive fluorescence features. Even more impressive was the fact that the anticancer properties of CBHAc extended the lives of tumor-bearing animals by decreasing the transition between epithelial and mesenchymal tissue (EMT). In this way, our cancer-targeting fluorescent agent opens up new avenues for theranostic precision medicine by providing a platform for intraoperative diagnostics as well as inhibition of cancer spread during surgery. A strategy was devised to confine ICG to the liver region directly close to a cancer, according to [16]. Real-time ICG fluorescence imaging was used to assess lymphatic flow in this study [17]. A subcutaneous injection of BJMC3879Luc2 cells, which have been shown to have a high incidence of lymph node metastasis, was employed as a model for testing. Lymph node metastases were examined histopathologically and with bioluminescent imaging after the animals had been sacrificed. NIR fluorescence imaging was used to assess lymphatic flow in a model with significant lymph node metastases. All injected mice had pathological metastases in their bilateral auxiliary, femoral, and para-aortic lymph nodes (100 percent). Using real-time NIR fluorescence imaging, the researchers discovered that the primary lymphatic vessels were still stained in the metastatic lymph nodes even after the cancer cells were inoculated. In the past, it was thought that obstruction of the principal lymphatic veins caused lymphatic flow to be altered through the bypass channel. After lymph node metastases, real-time ICG fluorescence imaging revealed no alterations in lymphatic flow. Colon cancer surgery may benefit from real-time ICG fluorescence imaging if the tumor has migrated to the lymph nodes. Colitis-related colon cancer was shown to be worsened by deletion of cGAS in mice [18]. For whatever reason, mice missing the cGAS gene or the type I interferon receptor were more vulnerable to CAC infection than mice with normal copies of either of these genes. Intestinal stem cells show a high level of cGAS, but not STING. This led to a loss of intestinal stem cells and to a decrease in intestinal barrier integrity after acute damage to the gut caused by dextran sodium sulphate (DSS). When cGAS was lost, inflammation was worsened, and STAT3 was activated, which resulted in an increase in intestinal epithelial cell proliferation. Tumor-associated myeloid-derived suppressive cells proliferated more abundantly in mice missing cGAS, and these cells demonstrated heightened Th17 differentiation, although their production of interleukin-10 (IL-10) was decreased. These findings show that cGAS protects the integrity of the intestinal mucosa in order to inhibit the growth of CAC. To treat cells inducible by TGF-, researchers utilized TRKIs SB431542 and LY2109761. Luciferase action was increased 5.24 times in CT26 and MC38 driven cells, but only minimally in MC38 cells missing Smad4. TGF-induced bioluminescence action was decreased by SB431542 treatment of mice for a short period of time [19]. RH was shown to have a wide range of cytotoxic properties, as demonstrated by [20] in CCD-18co, a cell line derived from normal human colon fibroblasts; RH was shown to be less hazardous. HCT 116's morphological and biochemical alterations were shown to be triggered by RH in cell death investigations. Multiple prosurvival proteins were downregulated at the protein level, whereas ROS, caspase-3/7, and TRAIL-R2 expressions were all increased in HCT 116. RH treatment of HCT 116 resulted in a substantial decrease in invasion, migration, and colony formation. Isoledene and elemene were found to be the most common chemicals in the GC–MS and HPLC analyses. In a xenograft model, RH was shown to be very effective in preventing tumor growth. RH has the potential to be an inexpensive anticolon cancer naturaceutical, according to these studies. In order to learn more about how the OLR1/c-MYC/SULT2B1 axis influences colon tumor cell proliferation and chemoresistance, this study [21] was undertaken. The next step was to use LoVo cells to perform ectopic expression and knockdown tests. MTS assays and clone creation were used to measure cell growth. Extracellular acidification and glucose absorption and lactate generation were assessed to determine glycolytic metabolism. ATP/ADP ratio was also calculated, and GLUT1 and LDHA expression was evaluated. As a result, c-MYC may be downregulated, reducing SULT2B1 expression and so inhibiting colon cancer cell growth and chemoresistance

It was shown that colitis-associated colon cancer (CAC) may be prevented by a combination of three probiotics known as a Bornlisy- (BO-) cocktail [22]. Tumor burden was reduced in CAC mice treated with BO compared to control mice. In vitro, BO also suppressed the growth and spread of tumor tissues. In addition, by reducing glycolysis, BO slowed cell growth. In the CAC mice, activating glycolysis abolished the protective effect of BO. GPR43 was activated mechanically by BO injection, which led to a reduction in glucose metabolism as a result of the PLC-PKC-ERK pathway. These findings imply that BO might be used as an intervention technique for cancer treatment, whereas GPR43 is a possible target receptor for BO therapy. Reference [23] found that the camptothecin analogue FL118 has antitumor action on a broad spectrum of malignancies, although the molecular mechanism behind its antitumor activity is still a mystery. Some researchers think that microRNAs, or “miRNAs,” are critical to human malignancy because they play a role in the growth of tumor, as well as the cancer-suppressive effect of natural and synthetic substances. miR-155, previously identified as an oncogenic miRNA in colorectal cancer, was shown to be considerably downregulated following FL118 therapy, according to our prior research. Apoptosis, cell viability, cell mobility, and cell proliferation were all reduced by FL118 in the colon cancer cell lines studied. FL118 substantially (P0.05) decreased miR-155 levels in vivo and in vitro.

## 3. Methodology Used

The data of mice is collected. The reagents and materials utilized for the analysis are examined. The extracts are prepared by using the combination of Chinese herbs such as Astragalus membranaceus and Curcuma zedoaria. The viability assay of the cell and transwell assay are evaluated. Further, the Western blot analysis is performed. Finally, the RNA purification, cDNA synthesis, and quantitative real-time PCR are determined. The statistical analysis is assessed, and it shows the potential impact and mechanism of astragalus and curcumin (AC) in the treatment of colon cancer, providing the insight into how to effectively use it.  Figure 1 represents the schematic representation of the suggested methodology.

### 3.1. Data Collection

The research employed SPF quality BALB/c adult mice (*n* = 125, 35 weeks old, mass 20.2 g) at Qinglongshan Livestock Breeding Farms, Jiangning District, Nanjing City, rodent models licence number SCXK (Su) 20170001. Mice were housed in a warm and humidity-controlled setting at Nanjing University of Chinese Medicine's Experimental Animal Center (Nanjing, Jiangsu, China). All animal experimentation has been authorised by the Ethics Committee in line with the National Institute of Health's Guide for the Clinical and Laboratory Standards Institute Animals of Nanjing University of Traditional Chinese Medicine (Nanjing, China). Five male C57Bl/6J mice, 1.5 months old and weighing between 20 and 25 g, were divided into groups and given weekly intraperitoneal injections or oral administrations of diluted Curcuma zedoaria dosages. Controls received dilutions of the extraction liquid at the same concentrations as the experimental groups. Curcuma zedoaria, diluted in water, was given to the other groups in two diverse concentrations. Every two weeks, the animals' weights were recorded, and heparin-infused blood was drawn from the venous retroorbital plexus (5,000 UI, Roche). Differential leukocyte counts were determined by spreading out small amounts of blood on glass slides, fixing them in a solution of methanol for five minutes, drying them, and then staining them with Giemsa (1 : 4) (Merck, Germany). Red blood cell suspension (1 : 10) was diluted with saline and stained with 1 : 10,000 total leukocytes. The animals were killed and necropsied after three months for oral route therapy and two months for intraperitoneal therapy, and the peritoneum cells were then washed with 2 mL of chilled PBS. Total resident cells in the peritoneal exudate were counted in Malassez chambers after it was collected. A microscope was used to count and evaluate the various kinds of leukocytes that had been deposited on glass slides. When the findings of the Curcuma zedoaria therapy were contrasted with those of the control group, a statistical analysis was performed. Data were summarized as the mean standard deviation (SD) for each group [24].

### 3.2. Reagents and Materials

FuHeng Biology provides us with HCT116 cells for our research (Shanghai, China). China's Sino Biological provided the CXCR4-overexpressing vector (MG50621-UT). WAY-262611 and SB 216763 were acquired from MedChemExpress China, while Astragalus membranaceus (HQ) and Curcuma zedoaria (EZ) were obtained from Jiangsu Province Hospital of TCM, respectively. Sigma-Aldrich supplied the rest of the required agents.

### 3.3. Cell Line and Cell Culture

HCT116 were cultured at 37°C using 5% CO_2_ and 95% oxygen in mixed medium containing 10% FBS, 100 g/mL ampicillin, and 100 g/mL streptomycin. HCT116 colon tumor tissues were cultivated at 37°C with 5% CO_2_ in RPMI-1640 media enriched with 10% FBS, 100 units/mL penicillin, 100 g/mL streptomycin, and 2 m ML glutamine. Once they achieved 70 to 80 percent convergence, cells were perfused with 0.25 percent trypsin/0.02% EDTA. The cells retrieved from freezing sources passed their maximal transit duration in very little than ten months. In the assays, logarithmic-phase lymphocytes were employed.

In the in vivo testing, male BALB/c mice with a bodyweight of 18–20 grams were used. Mice were supplied according to the livestock company's guidelines and housed in a pathogen-free setting with temperature and moisture controls. All animal testing were approved by the Institute of Animal Care and Use Committee at Shanghai University of Traditional Chinese Medicine in accordance with the International Standards of Animal Welfare (approval number: SYXK, Shanghai, 2013-0055).

In order to create the orthotropic HCT116 xenograft model, the following steps were taken: HCT116 cells were removed from the flask and diluted to 10 × 10^7^ mL^−1^ in growth media. The right auxiliary area of each of the five mice was injected subcutaneously with 200 L of cell suspension. Tumors extracted from the subcutaneous xenograft were split into pieces and implanted under the skin in the auxiliary area for the next-generation tumor mode after two weeks. To create the orthotopic xenograft model, researchers reportedly utilized tumors from the third subcutaneous generation. Subcutaneous tumors were collected and chopped into 1.5-millimeter pieces, nude mice were sedated, and the abdomen was disinfected with iodine and alcohol. The intestine's caecum was externalized by a tiny incision in the midline. Amyxis was used to remove serosa from the area where tumor parts were to be inserted. Medical adhesive was then used to secure the tumor fragments to the caecum wall. The abdominal wall was closed using surgical sutures after the intestine was reinserted into the abdominal cavity. Then, the animals were housed in a sterile environment.'

### 3.4. Preparation of Extracts of Astragalus membranaceus and Curcuma zedoaria

We employed three different concentrations of HQ and EZ, each extracted for one hour in 100°C water. Ten milligrams of crude medicines per litre was added to the solution. After cooling, the solution was centrifuged at 12000 × g for 10 minutes before the germs were removed using a 0.22 m filter. Afterward, the filtered solution was separated and kept at -20 degrees Celsius. Weight per millilitre is a measure of the amount of crude medicines in the solution. In September of 2012, Curcuma zedoaria was discovered in the Chinese region of Guangxi. They were sent to the Zhejiang Chinese Medical University's First Affiliated Hospital. The herbarium specimens validated the plant's identify by comparing its morphology to the specimens. There were 40 meshes of particle size reduction on the sample before it was ready for analysis. In a 100 mL flask containing 400 mL of 70 percent ethanol, the sample (40 grams) was weighed correctly and soaked overnight. Heating reflux was used twice to remove the sample. A residue was formed whenever the alcohol extract was obtained and condensed at low pressure. Then, petroleum ether was used to remove the remaining residue. To get the dried petroleum ether extracts, rotary evaporators were used to dry the ether extracts from petroleum. To make a 10 mg/mL stock solution, the five mg of petroleum ether extracts was dissolved in 500 L of DMSO. It was kept at a temperature of 20°C until it was required to be used. Cancer cell multiplication in vitro and cancer development in mice structures were both suppressed by the TCM herb curcumin, which is often used in cancer treatment because of its antibacterial anti-inflammatory and antiproliferative properties.  Figure 2 illustrates the broad methodologies used to test the anticancer activity of medicinal plant extracts from Astragalus membranaceus and Curcuma zedoaria in vitro and in mice.

To treat a broad range of illnesses and bodily dysfunctions, traditional Chinese medicine (TCM) often incorporates Astragalus membranaceus, an important medicinal plant, into its herbal preparations. Recent clinical trials have focused on the herb's chemical ingredients and the possibility of using them to treat inflammatory illnesses and malignancies. For patients using other traditional medications at the same time, therapy with astragalus has shown considerable improvement in the harmful effects (e.g., immunosuppressants and cancer chemotherapeutics). In Astragalus membranaceus, the most important polysaccharides, flavonoids, and saponins are present in the plant. Antioxidant, anti-inflammatory, and anticancer properties of Astragalus membranaceus are the primary focus of current usage. An investigation on the biological characteristics of Astragalus membranaceus and its primary ingredients was conducted. A new Astragalus saponin extract termed AST has been shown to have anticancer properties in the treatment of several gastrointestinal malignancies. Anti-inflammatory and anticancer properties of Astragalus herb and AST include modulation of numerous cancer signaling pathways and interaction with particular transcription molecules. A better treatment plan for inflammatory disorders and gut malignancies might benefit from this knowledge, which could lead to the development of innovative target-specific and effective therapeutic medicines that are free of substantial systemic adverse effects. TCM (traditional Chinese medicine) uses the dried root of Astragalus membranaceus (AM). Numerous studies have shown that AM has a broad area of biological properties, comprising of cardioprotective immunomodulatory, anti-inflammatory, and anticancer. Colon, breast, liver, hepatocellular, gastric, prostate, and cervical human tumor tissues in vitro were significantly inhibited by AM. The cancers of the colon and breast were also suppressed by AM.

Cancer is usually treated with cytotoxic medicines, radiation, chemotherapeutic, and surgery as a routine treatment. Traditional remedies, on the other hand, have garnered considerable attention in recent times. Herbal medicines are beneficial against colon cancer, with a focus on bioactive substances and fundamental mechanisms of action. The following Table 1 contains some of the available herbal medicines.

### 3.5. Cell Viability Assay

After 12 hours of treatment with HQEZ, 5 × 10^3^ cells/well HCT116 were plated in 96-well plates. The CCK8 test, as instructed in the user handbook, was used to determine cell viability after 24 hours. It was then cultivated for another hour before the optical density of CCK8 was calculated on an MFP microplate reader at the wavelength of 450 nanometers. The following equation was used to get the proliferation inhibition rate: one-OD-treated/OD‐controlled = 100%.

### 3.6. Transwell Assay

24 well transwell chambers were filled with 1 percent FBS and 1 × 10^5^ cells/well HCT116 (Costar). 50 L Matrigel was applied to the top region of polycarbonate filters with 8 mm pore sizes and left uncoated or applied. It was decided to use culture media that included 10% FBS in the lower chambers. It took 48 hours to cultivate the cells. To stop cell migration or invasion, the cells were removed from the upper chambers, dyed with crystal violet, and then discarded.

### 3.7. Western Blot Analysis

As previously stated, the examination of Western bolts was carried out as indicated. Here are the main antibodies: CXCR4 rabbit antiserum, rabbit antiserum against E cadherin, rabbit antiserum against N cadherin, rabbit antiserum against Vimentin, rabbit anti-catenin, rabbit antiserum against Myc, rabbit antiserum against cyclin D1, and rabbit antiserum against p-catenin. We employed mouse anti-GAPDH as an internal control, together with mouse anti-actin in order to boost the chemiluminescence detection process. The count of tissues that reached the bottom region of the filter was counted in five random fields per filter.

### 3.8. Precise Real-Time PCR, RNA Isolation, and cDNA Transcription

The HCT116 cells were plated at a density of 5 × 10^5^ cells/well in 6-well plates and then treated with HQEZ for 12 hours. Total RNA was isolated using Trizol after 24 hours, as per the methodology outlined in the text. Additionally, cDNA was generated using the M-MuLV First-Strand cDNA Synthesis Kit.

As part of our study, we used Sangon Biotech's B630004 qPCR Mastermix (Shanghai Co., Ltd. China) to run qPCRs in triplicate. The Ct technique was used to measure and normalise the expression of the target mRNA to -actin expression. The primers that were utilized are shown in Table 2.

## 4. Results and Discussion

### 4.1. Statistical Analysis

At least 3 distinct investigations were performed out. To summarise all of the data, standard deviations are utilized. The significance level was determined using the Student *t* test, with a *p* value of 0.05 determined largely.

#### 4.1.1. Cell Viability

Colorectal cells are inhibited by HQEZ. HCT116 cell viability was decreased dose-dependently by the CCK8 test after 24 hours of incubation with HQEZ, and extracts from the combination of HQ and EZ (2 : 1, weigh proportion) inhibited colorectal cells most effectively (Figures 3 and 4). These findings suggested that high doses of HQEZ might directly trigger apoptosis in colorectal cancer cells whereas low doses of HQEZ inhibited the cells' viability. We used HPLC to examine the chemical contents of the extraction of HQEZ to ensure that the extraction technique worked properly. It was observed that the process of heating up HQ and EZ combined resulted in a higher concentration of the active ingredients Astragaloside I, Astragaloside II, and Calycosin as well as the ability to trace the batches of pharmaceuticals.

#### 4.1.2. Metastasis Ability of Colorectal Cancer

Colorectal cancer cells' ability to spread is reduced by HQEZ. However, HQEZ is often used in adjuvant treatment to prevent colon tumor metastases and lengthen the lives of patients, not to inhibit cell viability, promote apoptosis, or halt the cell cycle. HQEZ is administered at a modest dosage in the clinic; thus, our research focused on how HQEZ affects colorectal cells' potential to metastasize. In vitro migration of HCT116 cells was dramatically reduced by HQEZ in a migration experiment (Figure 5). In vitro invasion assays also showed that HQEZ dramatically inhibited HCT116's capacity to invade in vitro (Figure 5). HQEZ was shown to inhibit colorectal cell metastasis at concentrations lower than those required to cause apoptosis or cell cycle arrest. Colorectal cancer cells' capacity to spread may be reduced by HQEZ, regardless of the extent of cell damage.

#### 4.1.3. Reduced EMT, CXCR4, and *β*-Catenin Signals Are Associated with the Inhibition of HQEZ on Colon Tumor Tissues

Liver metastasis is a common feature of colon tumor, and it is thought that CXCR4 expressed on colon tumor tissues reacts to CXCL12 generated from the liver, causing directed metastasis. The expression of CXCR4 in HCT116 was evaluated following the administration of HQEZ, and it was shown to be lowered, as shown in Figure 6. As a result, we hypothesized that HQEZ's suppression of CXCR4 would result in a reduction in HCT116's metastatic potential, particularly in the liver. *β*-Catenin, a critical component of the Wnt/*β*-catenin pathway, which is involved in cancer metastasis, has been linked to CXCR4 activation and has been shown to alter the EMT signaling pathway. *β*-Catenin was dramatically reduced after administration of HQEZ (Figure 7). It implied that the HQEZ impact should be related to the loss function of *β*-catenin and its downstream signal. The administration of HQEZ suppressed the CXCR4, *β*-catenin, and EMT signaling pathways, all of which are connected to one another; the interaction between these signaling routes and HQEZ should be investigated further.

#### 4.1.4. *β*-Catenin Was the Key Component Associated with the Effect of HQEZ

The translation of *β*-catenin was seldom reduced following administration of HQEZ, whereas the transcription of CXCR4 was significantly reduced (Figures 8(a) and 8(b)).

As seen in Figures 8(a) and 8(b), administration of HQEZ had no effect on the mRNA level of 𝛽-catenin in HCT116.

WAY-262611, a -catenin activator, was administered to HCT116 when they were treated with HQEZ because we hypothesized that HQEZ impacted 𝛽-catenin at a posttranscriptional level. In HCT116 treated with HQEZ, WAY-262611 (0.5 M) restored the expression of -catenin as well as the metastatic ability, EMT signal, and CXCR4 expression (Figures 9 and 10). HQEZ must enhance the phosphorylation of -catenin, only with degradation of -catenin lowering the transcription of genes related, such as EMT signaling pathway components as well as other features of metastatic.

#### 4.1.5. Astragalus, Curcuma, or Mixed Solution Displayed Diverse Effects on the HCT Cells

However, the combination of Curcuma and CXCR4 lowered the expression of CXCR4 in the 𝛽-catenin and c-MYC (Figure 11) compared to Curcuma alone.

## 5. Conclusion

Ancient Chinese treatment, Astragalus membranaceus, is commonly utilized in tumor treatment Astragalus membranaceus is suggested to improve immune function in tumor sufferers, and several natural factors from the plant promoted chemosensitivity or directly suppressed tumor cells. Astragalus membranaceus also defends sufferers from liver and nervous harm throughout chemotherapy, particularly from platinum-based toxicity. Curcuma zedoaria is another ancient Chinese treatment that is commonly combined with Astragalus membranaceus and has cytotoxic and tumor-inhibiting qualities. Researchers used water to retrieve Astragalus membranaceus and Curcuma zedoaria, which is a widespread use in medical. Researchers discovered that the retrieval was lethal at large levels and protected metastasis at less concentrations. Decreased metastasis is crucial in adjuvant therapies, and ancient Chinese remedies ensure that sufferers live longer, which would be partially due to the antimetastasis impact. Researchers found that HQEZ inhibited EMT and 𝛽-catenin in colorectal tumor cells, as well as reducing CXCR4 expression. HQEZ was first thought to repress CXCR4 in order to downregulate the Wnt/-catenin pathway, as reported in a previous research. While authors abundantly expressed CXCR4 in HCT116, they discovered no significant recovery of -catenin or the EMT system, but enhancement of the -catenin pathway recovered CXCR4, the EMT pathway, and invasive capabilities. Per some studies, the Wnt/-catenin pathway controls CXCR4, and essential components of the EMT process are also regulated in a Wnt/-catenin-related manner. Astragaloside IV, an effective element in Astragalus membranaceus, and -elemene, a main chemical in Curcuma zedoaria, are said to block the Wnt/-catenin pathway in investigations. These results are in line with previous research that suggests that inhibiting -catenin breakdown protects HCT116 against HQEZ. According to the results, HQEZ raised the phosphorylation of -catenin and subsequent degradation of -catenin, leading in the dysregulation of EMT signal and CXCR4, which were important in HQEZ's toxic activity on gastrointestinal tumor spreading potential. In conclusion, HQEZ inhibits the spread of colon tumor tissues in vitro by promoting the breakdown of 𝛽-catenin at a lower dosage. These findings reveal a potential action of conventional Chinese medicine in the treatment of colon cancers, paving the way for HQEZ to be employed as an adjuvant therapy for colon tumor individuals.

## Figures and Tables

**Figure 1:** Flow of the methodology used.

**Figure 2:** Anticancer activity of medicinal plant extracts.

**Figure 3:** Cell viability vs. milligram per millilitre HQEZ-induced HCT116.

**Figure 4:** Cell viability vs. milligrams per millilitre.

**Figure 5:** HQEZ reduced migration, despite the low dose that did not cause apoptosis.

**Figure 6:** Invasion of HCT116 cells, *p* < 0.05 compared with vehicle.

**Figure 7:** *p* < 0.05 when compared to vehicle exhibits HCT116 cell invasion.

**Figure 8:** (a, b) Effect of HQEZ on *β*-catenin.

**Figure 9:** WAY-262611, a possible promoter of -catenin, saved HCT116 cells against HQEZ.

**Figure 10:** Stabilization of *β*-catenin was essential to retain the potential to metastasize.

**Figure 11:** Curcuma or mixed solution but not the Astragalus reduced the invasion of HCT116.

**Table 1:** List of available herbal medicines.

S. No	Herbal name	Cell line	Concentration	Cellular effect
1	*Allium sativum*	HT-29	20, 50, 100 mg/mL	Apoptosis activation and apoptotic
2	*Punica granatum*	LS174	63.2 *μ*g/mL	Cytotoxic activity
3	*Olea europaea*	HT-29, HCT116,	NM	(i) Growth is stifled; (ii) movement and attack are stifled
4	*Piper betle*	HT-29 and HCT116	200.0 *μ*g/mL	Increased oxidative activity and activation of apoptosis
5	*Salvia ballotiflora*	CT26	6.76 *μ*g/mL	Cytotoxic activity
6	*Millingtonia hortensis*	RKO	200, 400, 800 *μ*g/mL	Antiproliferative effect
7	*Annona muricata*	HCT116, HT-29	11.43 ± 1.87 *μ*g/mL and 8.98 ± 1.24 *μ*g/mL	HT-29 and HCT116 cells are prevented from migrating and invading
8	*Suillus luteus*	HCT15	400 *μ*g/mL	An elevation in subcellular level of p-H2A.X, indicating damage to DNA
9	*Glehnia littoralis*	HT-29	50 mg/mL	Reduced appearance of the antiapoptotic Bcl-2 mRNA mediated apoptosis
10	*Hedyotis diffusa*	HT-29	400 mg/mL	Stimulate apoptosis in human CRC cells by inhibiting tumor cell development

**Table 2:** The primers that were utilized are listed.

Component	Forward	Reverse
*β*-Actin	AGCGAGCATCCCCCAAAGTT	GGGCACGAAGGCTCATCATT
*β*-Catenin	AAAGCGGCTGTTAGTCACTGG	CGAGTCATTGCATACTGTCCA

## Data Availability

On reasonable question, the authors will provide the dataset employed and/or analyzed even during present work.
